# Prediction Model for Infectious Disease Health Literacy Based on Synthetic Minority Oversampling Technique Algorithm

**DOI:** 10.1155/2022/8498159

**Published:** 2022-03-25

**Authors:** Rongsheng Zhou, Weihao Yin, Wenjin Li, Yingchun Wang, Jing Lu, Zhong Li, Xinxin Hu

**Affiliations:** ^1^The Third People's Hospital of Hefei, Hefei Third Clinical College of Anhui Medical University, Hefei 230022, China; ^2^Linyi Hospital of Traditional Chinese Medicine, Dezhou 251500, China

## Abstract

**Objective:**

Improving health literacy in infectious diseases is a direct manifestation of the solid advance in disease control and prevention. Our study is aimed at exploring applying synthetic minority oversampling technique (SMOTE) in the prediction assessment of whether residents and business employees have infectious disease health literacy.

**Methods:**

The Chinese resident infectious disease health literacy evaluation scale was used to investigate the associated variables. The screened variables were input variables and the presence or absence of infectious diseases health literacy as outcome variables. Logistic regression, random forest, and support vector machine (SVM) models were built in the data sets before and after treatment by the SMOTE algorithm, respectively, and the performance of the models was evaluated by receiver operating characteristic curves (ROC).

**Results:**

Logistic regression, random forest, and SVM achieved accuracies of 0.828, 0.612, and 0.654 before SMOTE algorithm processing, and the areas under the ROC curves (AUCs) of the three models were 0.754, 0.817, and 0.759, respectively. The accuracies were 0.938, 0.911, and 0.894 after SMOTE algorithm processing, and the AUCs of the three models were 0.913, 0.925, and 0.910, respectively.

**Conclusions:**

The random forest model based on the SMOTE has high application value in assessing whether residents versus enterprise employees have infectious disease health literacy.

## 1. Introduction

Infectious diseases are both transmissible and epidemic, posing a great danger to human health [1, 2]. With more developed transportation, logistics, and so on, the mobility and clustering of the population have increased, and the probability of all types of major infectious diseases spreading worldwide has risen dramatically. Once the infectious disease occurs, it quickly causes harm to the people's physical health and life safety. At the same time, it causes damage to social and personal properties even hinders social development [3, 4]. Health literacy is the ability of individuals to acquire or understand basic health information and services and use this information and services to make correct decisions to maintain and promote their health [5].

Infectious disease health literacy is part of health literacy. Health literacy and health status are closely linked. Low health literacy negatively impacts lifestyle, health service utilization, and adherence to interventions, resulting in high disease incidence and prevalence and poor disease outcomes [6]. The 2012 national health literacy surveillance results showed low health literacy among Chinese residents. Among the six categories of health problems, infectious disease prevention and treatment literacy was at a low level [7]. Infectious disease health literacy reflects residents' understanding and application to the initiation, prevention, and treatment of infectious diseases. The improvement of health literacy in infectious diseases is a direct manifestation of the solid advance in infectious disease control and prevention, and it is essential to control the spread of common infectious diseases, respond to large-scale infectious diseases, and enhance our ability to deal with public health crises [8]. High-level infectious disease health literacy among residents is both an objective need of the era and a powerful weapon to tackle the unknown challenges facing future infectious disease prevention and control efforts [9].

In this study, several machine learning prediction models were developed using data from the China health literacy evaluation scale for infectious diseases of residents. The models were based on the synthetic minority oversampling technique (SMOTE), and the prediction effects were compared. It is hoped that the low health literacy population will be screened to inform the development of targeted interventions through an established prediction model that predicts the health literacy status of an individual or a group.

## 2. Material and Methods

### 2.1. General Data

Considering this study as a stratified sampling study, the sample size was calculated according to the following formula:

(1) $$\begin{array}{c} N=\frac{u_{\alpha }^{2}\times p_{0}\left(1-p_{0}\right)}{\sigma^{2}}\times \text{deff}. \end{array}$$

According to the 2014 analysis of health literacy survey on prevention of infectious diseases among urban and rural residents of Hefei, the health literacy level of infectious diseases among urban and rural residents of Hefei is 49.4%. Using this as a reference, *P* = 0.494, relative allowable error *r* = 10%, then absolute allowable error =10% × 49.4% = 0.0494, calculated sample size of 950 participants based on 95%CI = 1.96, design efficiency deff = 1.5.

### 2.2. Study Subjects

The study subjects were residents and enterprise employees in the Jiakai District of Hefei City, and the questionnaire release time was from February 5, 2020, to February 12, 2020. In this investigation, 1900 questionnaires were issued cumulatively, and 1874 were returned, and the effective rate of the questionnaire was 98.63%.

### 2.3. Research Method

The health literacy evaluation scale for infectious diseases among Chinese residents was used, and the first part of the scale consists of 22 items [10].

The health literacy evaluation scale for infectious diseases among Chinese residents was used. The first part of the scale consists of 22 items belonging to four dimensions: F1: basic knowledge and concept of infectious diseases (seven items, which mainly examine the individual's basic knowledge and concept on the infectious sources, transmission routes, and susceptible populations of common infectious diseases); F2: prevention of infectious diseases (7 entries that primarily examine an individual's knowledge of common infectious disease precautions); F3: management and treatment of infectious diseases (4 entries, mainly looking at the mastery of management and treatment of common infectious diseases); and F4: recognition of infectious disease (4 entries that primarily examine an individual's ability to discern common infectious agents and symptoms). Cronbach's *a* for the four dimensions was 0.654, 0.673, 0.562, and 0.638, with a construct validity of 0.8 for each item. The second part of the Chinese health literacy assessment scale for infectious diseases of residents, which consists of 6 items with genera measuring separate dimensions of responders' cognitive abilities, was not included in the analysis. F1 was set as the exogenous dependent latent variable (not affected by the other latent variables), based on expertise in infectious disease health literacy; F2, F3, and F4 were set as the internal dependent latent variables (influenced by other latent variables). The magnitude of the mutual effect between the four latent variables of the China health literacy assessment scale for infectious diseases among residents is the effect value. The direct effect between the two latent variables is termed the immediate effect. The effect produced through an intermediate variable is the indirect effect, and the sum of the immediate effect versus the indirect effect is the total effect. The flow chart of scale analysis is shown in Figure 1.

### 2.4. Model Building

Python 3.7 software was used to establish the prediction model. Calling train_test_split in sklearn.model_selection and randomly split the data set into four parts: the first 3/4 as the training set was used to build the model, and the remaining 1/4 as the test set was used to evaluate the model performance. Logistic regression models were built in the training set with place of residence, educational level, occupational class, whether they had healthcare related work and monthly household income as input variables, and whether they had health literacy as predictor outcome, respectively, after univariate screening with random forest and support vector machine (SVM). Most machine learning algorithms' classification accuracy decreases substantially when the data become imbalanced [11–13]. Thus, the models were then applied in the test set to assess whether residents and business staff possess infectious disease health literacy.

SMOTE algorithm is an improved scheme based on the random oversampling algorithm (Figure 2). Because random oversampling adopts the strategy of simply copying samples to increase a few samples, it is easy to produce the problem of model overfitting, even if the information learned by the model is too specific and not general [14]. The basic idea of the SMOTE algorithm is to analyze a small number of samples, synthesize new samples, and add them to the data set according to the small number of samples, as shown in the figure below. The algorithm process is as follows:

1. For each sample *x* in the minority class, the distance from it to all samples in the minority class sample set is calculated by taking the Euclidean distance as the standard, and its *k*-nearest neighbor is obtained
2. A sampling ratio is set according to the sample imbalance ratio to determine the sampling magnification n. For each minority sample *x*, several samples are randomly selected from its *k*-nearest neighbors, assuming that the selected nearest neighbor is *x*_*n*_
3. For each randomly selected nearest neighbor *x*_*n*_, a new sample is constructed with the original sample according to the following:

(2) $$\begin{array}{c} x_{\text{new}}=x+\mathrm{rand}\left(0,1\right)\times \left(\tilde{x}-x\right) \end{array}$$

To improve the classification accuracy of machine learning, this study again adopted the synthetic minority class oversampling technique for repeated sampling, so that the data tended to be balanced. This process employs R3.7, the software calls the synthetic minority oversampling technique (SMOTE) package, settings perc.over = 600, perc.under = 200, to generate new data. The previous modeling process was repeated in this new data one more time.

### 2.5. Statistical Processing

Model establishment and evaluation were implemented through the software Python 3.7: logistic regression model was built by applying logistic regression in sklearn.linear_model; random forest models were built applying the randomforestclassifier in sklearn.ensemble, n_estimators = 100; SVM model building by applying the SVC in sklearn.svm, *C* = 100, gamma = 0.001.

## 3. Result

### 3.1. Input Variable Filtering

Univariate screening of independent variables was performed prior to model building: a logistic regression model was constructed using the presence or absence of health literacy as the dependent variable and the nine factors included in the questionnaire as independent variables, with a test level of 0.05, and gender, education level, and age were screened out as input variables. Specific results are shown in Table 1.

### 3.2. Comparison of Performance of Each Classification Model on Raw Data without the SMOTE Algorithm

Logistic regression, random forest, and SVM models were trained on the training data set after one hot coding of the univariate filtered independent variables as input variables, with health literacy as the outcome variable or not. The random forest model was subjected to a grid search optimal n_estimators taken 100. The SVM model was subjected to a grid search optimal *C* taken 100 and gamma taken 0.001. Tests were performed in a test data set with the real situation. The precision of all three models exceeded 90%, but several other metrics were low, especially recall and *f*-scores. The greater the curve areas under the ROC curves (AUCs) in the receiver operating characteristic (ROC) plot indicates better model performance, and the higher the ROC curve for the random forest model than for the logistic and SVM models. Specific results are shown in Table 2 and Figure 3.

### 3.3. Comparison of Performance of Each Classification Model on Data Processed by the SMOTE Algorithm

After the raw data were processed with the SMOTE algorithm, the new data set was used with the same method to build a model and compare the performance. The precision of all three models decreased, but each of the other indexes increased significantly. The random forest model had a higher recall, *f*-scores, accuracy, and AUC than the other two models, and the specific results are shown in Table 3 and Figure 4.

## 4. Discussion

Health literacy is an essential measure of the state's basic level of public service and people's health. It is also considered a key factor influencing the prevention and management of chronic diseases [15]. Low-level health literacy severely negatively impacts overall national health and the national health system. It has become a severe public health problem that has received extensive attention [16, 17]. Many factors associated with low-level health literacy are also associated with health disparities and may influence health outcomes. Infectious disease health literacy is an essential component of individual health literacy, which can be used both as a basis for developing regional infectious disease control and for assessing the outcomes of infectious disease control efforts [18, 19]. In this study, we trained three machine learning models based on the original data and the balanced data processed by the SMOTE algorithm, respectively, and compared their performances through the mediation results of the communicable diseases health literacy evaluation scale for Chinese residents, and finally proposed an effective prediction model to provide the basis for implementing measures such as monitoring and evaluation of infectious diseases health literacy.

Imbalanced sample refers to the fact that in classification problems; there are classes in the training sample with particularly large sample numbers and some classes with particularly small sample numbers [20]. When there is class imbalance in the data set, it can have a large impact on the classification sensitivity of machine learning. In fact, in the real world, data are unbalanced [21]. The class imbalance problem has a wide range of applications in many ways. In all described uses, minority classes have high sensitivity and its information is the goal. However, classification algorithms are attracted to most classes and ignore a few. Therefore, their predictions for minority populations are mostly less accurate.

SMOTE is a oversampling technique for imbalanced data sets, which is considered as a preprocessing step of learning algorithms and an effective and common method to deal with class imbalance [20, 22, 23]. After SMOTE resampling of the original data to balance the data, logistic regression, random forest, and SVM models were trained again on the new data set. The results showed that the random forest model had higher performance than the other two models in the prediction of infectious disease health literacy for both residents and business employees, which can provide some credit for the prediction of infectious disease health literacy as well as the later delivery of interventions. Compared with traditional logistic regression methods, random forests balance sample error through random feature selection and are more convincing results than logistic models fitted with only a single test sample. SMOTE is considered an effective and common method to deal with class imbalance，but it also increases the cycle, which resulting in the decrease of computing performance [14, 22].

## 5. Conclusion

In summary, it is feasible to continuously improve residents' basic knowledge and concepts of infectious diseases, recognition, and prevention skills of infectious diseases by means of health education and health promotion approaches, which will lead to improved levels of infectious disease management and treatment. The random forest model based on the SMOTE has high application value in assessing whether residents versus enterprise employees have infectious disease health literacy.

## Figures and Tables

**Figure 1:** Flow chart of scale analysis.

**Figure 2:** Schematic diagram of SMOTE algorithm.

**Figure 3:** ROC curves of three classification models applied to the raw data.

**Figure 4:** ROC curve of three classification models applied to data processed by the SMOTE algorithm.

**Table 1:** Univariate analysis of health literacy and health behavior of residents and employees of enterprises.

Items	Resident		Enterprise staff	
	Health literacy	Health literacy	Health literacy	Health literacy
Gender				
Male	36.33 ± 4.70	11.19 ± 1.65	36.42 ± 4.75	11.23 ± 1.66
Female	36.91 ± 4.49	11.33 ± 1.66	36.87 ± 4.41	11.27 ± 1.63
*t*	1.309	0.898	0.972	0.245
*P*	0.191	0.370	0.331	0.806
Degree of education				
Junior high school and below	33.00 ± 2.95	9.33 ± 0.95	33.29 ± 3.31	9.47 ± 1.10
Senior high school/vocational high school/technical secondary school	35.31 ± 3.11	11.33 ± 0.95	35.50 ± 3.39	11.34 ± 1.00
Junior college	38.31 ± 4.65	11.66 ± 0.25	38.27 ± 4.63	11.65 ± 1.24
Undergraduate	39.00 ± 4.35	13.00 ± 0.82	39.30 ± 4.27	12.88 ± 0.89
Postgraduate	43.33 ± 3.40	14.00 ± 0.84	43.53 ± 3.41	14.00 ± 0.82
*F*	67.406	217.531	65.143	196.757
*P*	<0.001	<0.001	<0.001	<0.001
Age				
16~20 years old	33.10 ± 2.98	9.48 ± 1.06	33.35 ± 2.82	9.46 ± 0.90
20~30 years old	35.59 ± 3.55	11.33 ± 1.22	34.87 ± 3.75	10.82 ± 1.52
30~40 years old	38.54 ± 4.64	11.88 ± 1.31	38.51 ± 4.70	11.84 ± 1.28
40~50 years old	39.82 ± 4.60	13.22 ± 0.96	39.25 ± 4.41	12.68 ± 1.28
>50 years old	34.51 ± 3.68	10.38 ± 1.43	35.85 ± 5.31	11.27 ± 2.10
*F*	47.862	107.497	28.792	48.625
*P*	<0.001	0.037	<0.001	<0.001

**Table 2:** Performance comparison of the 3 classification models applied to raw data.

Model	Recall	Accuracy rates	f-scores	Precision	AUC
Logistic	0.291	0.828	0.431	0.936	0.754
Random forest	0.349	0.612	0.448	0.932	0.817
SVM	0.419	0.654	0.497	0.938	0.759

**Table 3:** Performance comparison of 3 classification models applied to data processed by SMOTE algorithm.

Model	Recall	Accuracy rates	*f*-scores	Precision	AUC
Logistic	0.608	0.938	0.739	0.816	0.913
Random forest	0.732	0.911	0.817	0.855	0.925
SVM	0.741	0.894	0.806	0.851	0.910

## Data Availability

The data presented in this study are available on request from the corresponding author.
